# HPLC Fingerprint Analysis of *Rana chensinensis* Eggs from Different Habitats and Their Antitussive Effect

**DOI:** 10.1155/2022/9229970

**Published:** 2022-10-22

**Authors:** Yang Xu, Fangfei Xu, Yuejie Wang, Xu Wang, Huiwei Bao

**Affiliations:** ^1^College of Pharmacy, Baicheng Medical College, Baicheng 137000, Jilin, China; ^2^Plant Chemistry Laboratory, Chinese Institute of Jilin Ginseng, Changchun, China; ^3^College of Pharmacy, Changchun University of Chinese Medicine, Changchun 130117, Jilin, China

## Abstract

In this paper, a novel fingerprint method was established for the quality control of *Rana chensinensis* eggs (RE) by high-performance liquid chromatography (HPLC). Cluster analysis and principal component analysis were performed. Besides, the antitussive effect of RE was explored. The analysis was achieved on a Kromasil 100-5C_18_ (4.6 mm × 250 mm, 5 *μ*m) column by gradient elution using methanol-0.1% phosphoric acid solution as the mobile phase. The influence of RE on cough latent periods and cough times of mice was investigated via an ammonia cough-inducing experiment. The validated HPLC method was precise, reproducible, and stable. The HPLC fingerprints of 10 batches of RE samples displayed 31 well-resolved common peaks in the chromatogram. Three of these peaks were identified and assigned to 1-methyl hydantoin, estradiol, and 4-cholestene-3-one. The similarities of 10 batches of samples were more than 0.95. RE from different origins could be classified into three groups via SPSS 23.0 software, suggesting RE samples from various provinces (Jilin, Liaoning, and Heilongjiang) can be well distinguished via the established method. High dose and middle dose of the RE group can significantly prolong the cough latent periods of mice (*P* < 0.05 or *P* < 0.01) and inhibit the cough times of mice (*P* < 0.01), indicating RE had a good antitussive effect. HPLC fingerprint combined with multicomponent determination can be an efficient and useful method for monitoring the quality of RE. This study also provided a more comprehensive strategy for the quality evaluation of RE.

## 1. Introduction

*Rana chensinensis*, known as Hashima, belongs to *Rana* genus of Ranidae in Anura (amphibia) [1]. It is a kind of animal with precious medicinal and economic value. Oviductus ranae is the dry product of the oviduct of *Rana chensinensis*, which has the effects of tonifying the kidney and essence, nourishing yin, and moistening the lungs. Besides, Oviductus ranae (OR) is popular in folk as a tonic and a valuable traditional Chinese medicine [2, 3]. The eggs of *Rana chensinensis*(RE), a by-product, are usually abandoned in the processing of the Oviductus ranae collection [4]. However, research studies in recent years revealed that RE not only contains protein, amino acid, crude fat, vitamin, lecithin, estrogen, and other essential elements of the human body but also has good antifatigue, antioxidant, and immunity-regulating effects [5, 6]. With the improvement of understanding of RE, healthcare products such as oral liquid, soft capsules, and tablets of RE have been developed in the market at present [7].

Fingerprint of traditional Chinese medicine (TCM) is the specific chromatogram of TCM and Chinese patent medicine samples from different places and batches, which is established through reasonable analysis means after appropriate treatment [8, 9]. The fingerprint could provide a basis and foundation for the identification and quality control of TCM [10–12]. This method has been widely used in a variety of TCM and compound preparation nowadays [13]. The fingerprint of TCM can not only guarantee the authenticity, stability, and consistency of the samples but also meet the complexity and integrity characteristics of TCM [14]. It is a reliable, accurate, and comprehensive quality standard and quality evaluation method of TCM. Some common problems still existed in animal medicine so far, such as unclear species background, imperfect quality control, evaluation system, poor specificity of inspection, and identification technology [15].

There are many effective compounds in RE, of which 1-methyl hydantoin, estradiol, and 4-cholestene-3-one are representatives. 4-cholestene-3-one is a kind of steroid compound related to the antifatigue effect. Estradiol can regulate the hormones in vivo. 1-methyl hydantoin is the main antitussive and anti-inflammatory compound. At the same time, these three active compounds are also the main active related compounds in OR. Therefore, the simultaneous determination of these compounds is of great significance for the quality evaluation of RE. Therefore, high-performance liquid chromatography (HPLC) fingerprint and multicomponent determination of RE samples from 10 regions were performed in this study, which offers a reference for the identification and quality evaluation of this medicine as well.

According to the literature, several active ingredients in RE also exist in OR, such as 1-methyl hydantoin. 1-methyl hydantoin is an index compound of OR in Chinese Pharmacopoeia (2015 Edition), which is related to the antitussive and anti-inflammatory effects of OR. Therefore, our group deduces that RE may have the same antitussive effect as OR. This study can increase the new activity and application scope of RE.

## 2. Experimental

### 2.1. Chemicals and Reagents

1-methyl-hydantoin (batch number: 111836-201102) and estradiol (batch number: 100182-201205) were all purchased from China Pharmaceutical Biological Products Verification Institute (Beijing, China). 4-cholesten-3-one (batch number: S45539-479) was obtained from Sigma Company (USA). Methanol (Fisher, America) was of chromatographic grade. Phosphoric acid, ammonia water, and other reagents (Beijing Chemical Industry Factory) were of the analytical grade. Chuan Bei loquat ointment was obtained from Jingdu nianci'an Co., Ltd. Ultrapure water was acquired from Hangzhou Wahaha Co., Ltd.

### 2.2. Laboratory Animal

The Institute of Cancer Research (ICR) mice (SPF grade) were provided by Jilin Yisi Experimental Animal Co., Ltd. The production license no. of the mice described above was SCXK (Ji)-2016-0003, which was used by Changchun University of Traditional Chinese Medicine with the use license no. of SCXK (Ji)-2016-0017. Besides, the ethics number of laboratory animals was 2018245. These animals were all raised in the experimental animal center of Changchun University of Traditional Chinese Medicine. The mice were fed with pellet feed for rats and given free drinking water under a certain room temperature (20°C∼23°C) and humidity (44%∼57%). The pellet feed for rats (SPF grade) was supplied by Jilin Yisi Experimental Animal Co., Ltd.

### 2.3. Animal Materials

RE in northeast China were purchased from various TCM markets. RE were found to be the eggs of *Rana chensinensis*, which were identified by the associate professor (Jinglei Xiao) of the Changchun University of Chinese Medicine. The sources and batch numbers of the representative RE samples are shown in Table 1.

### 2.4. Instrumentation

Chromatographic analysis was performed on a Agilent 1260 high-performance liquid chromatography system (including quaternary low-pressure mixing pump, auto-sampler, column oven, 1100 diode array detector, and ChemStation workstation). The AB135-S electronic balance was purchased from Mettler Toledo International Co., Ltd. The KQ-250 ultrasonic cleaner was obtained from Kunshan Ultrasonic Instrument Co., Ltd. The R series rotatory evaporator was acquired from Shanghai Shenzhen Technology Co., Ltd. The YLS-8A multifunctional cough and asthma-inducing instrument was obtained from Jinan Yiyan Technology Development Co., Ltd.

### 2.5. Chromatographic Conditions

The simultaneous determination was carried out on Kromasil 100-5C_18_ (250 mm × 4.6 mm, 5 *μ*m) monitored at 215 nm. The injection volume was 5 *μ*L. The mobile phase was composed of methanol (A) and 0.1% phosphoric acid solution (B). The detailed gradient elution conditions are shown in Table 2.

### 2.6. Standard and Test Solution Preparation

An appropriate amount of 1-methyl hydantoin, estradiol, and 4-cholesten-3-one was weighted precisely, placed in different volumetric flasks, and dissolved and diluted with methanol to obtain standard solutions with the concentration of 1-methyl hydantoin at 65.0 *μ*g/mL, estradiol at 173.4 *μ*g/mL, and 4-cholestern-3-one at 333.2 *μ*g/mL, respectively. Subsequently, 1-methyl hydantoin standard solution (precise 0.1 mL), estradiol standard solution (precise 1 mL), and 4-cholesten-3-one standard solution (precise 1 mL) were taken and dissolved with methanol (final adjusted volume 10 mL) to obtain a mixed standard solution with the concentration of 1-methyl hydantoin at 0.65 *μ*g/mL, estradiol at 17.34 *μ*g/mL and 4-cholesten-3-one at 33.32 *μ*g/mL.

Approximately 2.5 g of finely ground RE was accurately weighed and placed in a conical flask with a stopper. Then, methanol (20 mL) was added into the conical flask and was ultrasonically (250 W, 40 kHz) extracted for 30 min. The methanol extracts were cooled and filtered after making up the deficiency. The sample was extracted three times together. Then, the extracts were combined and evaporated to dryness using a roller evaporator. Finally, the residue was redissolved with methanol (final adjusted volume 25 mL) and shaken well. The solution above was filtered through a 0.22 *μ*m microporous membrane filter, and the subsequent filtrate was collected as the test solution.

### 2.7. Method Validation of HPLC Fingerprint [16]

In order to obtain a stable HPLC fingerprint of RE for quality evaluation, the precision, stability, and repeatability of the proposed method were investigated. The RSDs of the RRT and RPA of each common peak were calculated, respectively.

The precision test was evaluated by injecting the mixed standard solution into HPLC six continuous times on the basis of the developed chromatographic conditions. The stability test was assessed by analyzing the same test solution (stored at room temperature) at 0, 2, 4, 8, 12, and 24 hours, respectively. A repeatability test was carried out by determination of six parallel test solutions of the RE sample with the same batch number (S4). Besides, retention time and chromatographic peak areas of each peak in chromatograms obtained in the above experiments were recorded. The RSDs of the RRT and RPA of each common peak were calculated, respectively.

### 2.8. Establishment of the HPLC Fingerprint

Ten batches of RE samples were taken, prepared into test solutions, and injected into the chromatogram for analysis to obtain chromatograms to be analyzed. Then, the recorded chromatograms were imported into the similarity evaluation system for the chromatographic fingerprint of TCM (2004A edition) for analysis to obtain the control chromatogram and HPLC superposed fingerprints of 10 batches of RE samples. The reference chromatogram of RE was generated using S1 as the reference chromatogram via the median method after multipoint correction. The width of the time window was set as 0.1.

### 2.9. Method Validation of Quantitative Determination [17]

#### 2.9.1. System Suitability Test

The mixed standard solution and test solution were injected into the chromatogram for analysis according to the developed chromatographic conditions, respectively.

#### 2.9.2. Calibration Curves

A mixed stock standard solution of 1-methyl hydantoin, estradiol, and 4-cholesten-3-one was prepared at 20.80 *μ*g/mL, 19.24 *μ*g/mL, and 99.00 *μ*g/mL, respectively. The mixed stock standard solutions (precisely 0.2 mL, 0.4 mL, 1.0 mL, 2.0 mL, 5.0 mL, and 10 mL) were placed in different 10 mL volumetric flasks and dissolved with methanol (adjusted to volume 10 mL), respectively, to obtain the standard serial working solutions. Subsequently, 5 *μ*L each of the working solutions was injected into the chromatogram for determination on the basis of proposed chromatographic conditions. The standard curve was drawn by using the chromatographic peak area (Y) as the vertical axis and the concentration of standard solutions (X) as abscissa. In addition, the mixed standard solution was diluted with methanol gradually. The limits of detection (LODs) and limits of quantification (LOQs) were determined by three times and ten times the signal-noise ratio, respectively.

#### 2.9.3. Repeatability

Six copies of RE samples (2.5 g) with the same batch number (S4) were weighed and prepared into six parallel test solutions. Subsequently, six test solutions were injected into the chromatogram for analysis, respectively. Besides, the peak areas and RSDs of the contents of these three compounds were recorded and calculated, respectively.

#### 2.9.4. Precision

The mixed standard solution was taken and injected into the chromatogram six continuous times in the light of the established chromatographic conditions, respectively. Besides, RSDs of peak areas of 1-methyl hydantoin, estradiol, and 4-cholesterin-3-one were calculated.

#### 2.9.5. Stability

5 *μ*L of the same test solution (stored at room temperature) was injected into the chromatogram at 0, 2, 4, 6, 8, and 12 hours for determination, respectively. The peak areas of each component were recorded, and RSDs of peak areas were calculated, respectively.

#### 2.9.6. Recovery Rate

Six copies of RE samples (1.25 g) with known contents were accurately weighed and placed in six different stoppered conical flasks, respectively. Then, 0.1 mL of 1-methyl hydantoin standard solution (0.1006 mg/mL), 0.1 mL of estradiol standard solution (0.0796 mg/mL), and 0.2 mL of 4-cholestene-3-one standard solution (0.606 mg/mL) were added into the six conical flasks above and prepared into test solutions, respectively. Finally, 5 *μ*L of the test solutions was taken and injected into the chromatogram for analysis. At the same time, peak areas of each analyte were recorded and recovery rates were calculated, respectively.

### 2.10. Quantitative Determination of Three Active Components in RE

Ten batches of RE samples were taken and prepared into test solutions, respectively. Then, the test solutions above were injected into the chromatogram for determination. Peak areas and contents of three various compounds were recorded and calculated by the external standard method, respectively.

### 2.11. Antitussive Effect of RE on Mice

The mice were divided into the model group, Chuan Bei loquat ointment group (5.85 ml/kg), a low dose of the RE group (0.5 g/kg), a middle dose of the RE group (1 g/kg), and a high dose of the RE group (1 g/kg) randomly. There were ten healthy mice in each group. The mice in each group were given intragastric administration according to the dose. The model group was given the same dose of distilled water. After continuous administration for 5 days, the mice of each group were placed in an ammonia cough-inducing device of YLS-8A multifunctional cough and asthma-inducing instrument. 50% ammonia was sprayed on the mice for 30 s at constant pressure. Subsequently, the first cough time and cough latent period were recorded. Meanwhile, the cough times within 3 minutes were recorded.

## 3. Results

### 3.1. Method Validation of HPLC Fingerprint

The precision test results of the HPLC fingerprint showed that RSDs of RRT and RPA were less than 1.02%, suggesting that this method was of good precision. The results of the repeatability test exhibited that RSDs of RRT and RPA were less than 2.17%, illustrating that this method had good repeatability. Furthermore, the stability results displayed that RSDs of RRT and RPA were less than 1.89%, which indicated that the test solution was stable within 24 hours.

### 3.2. Establishment of HPLC Fingerprint

The generated reference chromatogram is shown in Figure 1. A total of 31 well-resolved peaks were confirmed as common peaks in HPLC-superposed fingerprints (Figure 2) of 10 batches of samples. Chromatographic peak 29 was considered as a reference peak owing to moderate retention time, better resolution, large peak area, and good stability. Relative retention times (RRTs) and relative peak areas (RPAs) of each common peak were calculated for method validation. The results are displayed in Tables 3 and 4.

Three characteristic peaks in the HPLC chromatogram were attributed to 1-methyl hydantoin (peak 2), estradiol (peak 14), and 4-cholestene-3-one (peak 29) by comparing them with the chromatogram of mixed standard solution. The HPLC chromatograms of mixed standard solution and test solution of RE are displayed in Figure 3.

The similarity of 10 batches of RE samples was estimated by the evaluation system for chromatographic fingerprint of TCM (2004 A edition) using HPLC contrast chromatogram as reference [18]. The analysis results are shown in Table 5. It turned out that the similarities of all samples were more than 0.95, which suggested there was little difference among those samples. The quality of 10 batches of samples was of good stability.

The RE samples were analyzed by SPSS 20.0 software using the RPA of each common peak as a variable. In addition, hierarchical cluster analysis (HCA) was performed according to the Ward method of Euclidean distance hierarchical clustering method [19]. The analysis results are displayed in Figure 4. The results illustrated that 10 batches of samples were categorized into group 1 (S4, S5, S6, S7, S8, S9, and S10), group 2 (S1 and S2), and group 3 (S3) when Euclidean distance was set as 10. The HCA results demonstrated that the quality of RE was significantly influenced by different habitats and provinces. Therefore, HCA can be used for the identification and classification of RE from different provinces.

Principal component analysis (PCA) [19] was conducted by importing common peak areas of RE samples (10 batches) to SPSS 23.0 software in order to evaluate the qualities of RE from different habitats comprehensively. The eigenvalues of the correlation matrix and variance contribution rates of 10 batches of RE samples are calculated and exhibited in Table 6. Selecting eigenvalue > 1 as extracted criteria, the cumulative variance contribution rate of the first three principal components was 85.509%. In addition, the scree plot (Figure 5) clearly reflected the information trend represented by each principal compound, which was in accordance with the results in Table 6. The first three principal compounds can be used to characterize the HPLC fingerprint of RE basically. At the same time, the weight proportion of each principal component and the correlation coefficient of each common peak were analyzed in this study. The loading matrix results (Table 7) indicated that both three active compounds and other unknown compounds were involved in the quality expression as the main information. The information expression of peaks 2 (1-methyl hydantoin), 6, 7, 15, 18, 19, 20, 21, 22, 23, 25, 26, 27, 28, 29 (4-cholestene-3-one), and 30 were mainly reflected by principal compound (1). Besides, the information expression of peaks 1, 12, and 17 were mostly reflected by the principal compound (2). The information expression of peaks 10, 11, and 13 were chiefly reflected by the principal compound (3).

### 3.3. Method Validation of Quantitative Determination

As is displayed in Figure 3, the chromatographic peaks of the three compounds were well separated and the number of theoretical plates was more than 3,000. The results suggested that this method was of good system suitability. The regression equations of three active compounds are shown in Table 8, indicating that each analyte presented good linear relationships within their own determination ranges and good sensitivity under the developed chromatographic conditions. The precision RSDs of peak areas of 1-methyl hydantoin, estradiol, and 4-cholestene-3-one were 1.38%, 1.92%, and 1.63%, respectively, suggesting that the developed method was of high precision. The stability RSDs of peak areas of 1-methyl hydantoin, estradiol, and 4-cholestene-3-one were 1.19%, 1.88%, and 1.59%, respectively, proving that the test solution was stable within 12 hours. The RSDs of contents of 1-methyl hydantoin, estradiol, and 4-cholestene-3-one in the reproducibility test were 1.54%, 1.93%, and 1.78%, respectively, suggesting that the proposed method had good reproducibility. The mean recoveries of three analytes ranged from 98.90% to 99.10% with RSDs of 1.72% to 1.91%, as shown in Table 9. The results above indicated that this analytical method was of high accuracy.

### 3.4. Quantitative Determination of Three Active Compounds in RE

The developed method was applied for the simultaneous determination of three active compounds in RE. The contents of 1-methyl hydantoin, estradiol, and 4-cholestene-3-one ranged from 5.949 to 14.463 *μ*g/g, 5.615 to 13.653 *μ*g/g, and 52.611 to 147.602 *μ*g/g, respectively. The determination results are summed up in Table 10.

### 3.5. The Antitussive Effect of RE

Coughing occurred at different times in all administration groups. The cough latent periods and cough times of mice in different groups varied to some extent. Chuan Bei loquat ointment group and high dose and middle dose of the RE group can not only significantly prolong the cough latent periods of mice (*P* < 0.05 or *P* < 0.01) but also significantly inhibit the cough times of mice (*P* < 0.01). The results are displayed in Table 11. The results indicated that RE had a good antitussive effect.

## 4. Discussion

With the increasing demand for traditional Chinese medicine (TCM) and the strengthening of drug safety awareness, quality control of TCM is becoming more and more significant currently. The HPLC fingerprint, an effective quality control mode of TCM, has been unanimously recognized in the world due to its scientific theoretical basis [20]. The HPLC fingerprint can provide sufficient and reliable information even if the chromatographic peaks belong to unknown compounds, which can be applied to control the quality of TCM [21, 22].

Optimization of chromatographic conditions played an important role in the development of the HPLC fingerprint. Influence of different mobile phase systems (methanol-water, acetonitrile-water, methanol-0.1% phosphoric acid-water, methanol-0.2% phosphoric acid-water, acetonitrile-0.1% phosphoric acid-water, and acetonitrile-0.2% phosphoric acid-water) on separation effects of chromatographic peaks were investigated [23–25]. The results suggested that gradient elution of the methanol-0.1% phosphoric acid solution system could achieve better separation effects, good peak shape, and moderate retention time. Therefore, gradient elution of methanol-0.1% phosphoric acid solution was applied in this study. Besides, different detection wavelengths (215, 225, 267, 320, and 360 nm) were checked. Finally, the detection wavelength was confirmed as 215 nm. Since there were more chromatographic peaks under the wavelength above, this could meet the request of HPLC fingerprint study.

The HPLC fingerprint of RE established in this paper can reflect the specific and overall information of medicinal materials [26]. Three compounds (peak 2, 1-methyl hydantoin; peak 14, estradiol, and peak 29, 4-cholestene-3-one) were identified by comparing them with the HPLC chromatogram of the mixed standard solution. The similarity evaluation results showed that 10 batches of RE samples were of high similarity in general even though there were some differences between the qualities of each sample. Moreover, there was little difference between the RSDs of RRT of common peaks. However, the RSDs of RPA had certain distinctions. The results indicated that although the composition of RE samples from different places maintained the same, there was some diversity among the contents [27, 28]. RE samples from various provinces (Jilin, Liaoning, and Heilongjiang) can be well distinguished via the established HPLC fingerprint, which further suggested that the composition change of RE was affected by environmental factors.

The results of the determination displayed that the content of each of the three active compounds in the RE from Xinbin of LiaoNing province was higher than in other origins, except for Fusong in Jilin province. Contents of these compounds in RE from LiaoNing province were higher than those in most samples of Jilin and Heilongjiang provinces. In addition, the contents of these compounds in RE from Jilin province were higher than those in the majority of samples from Heilongjiang province. The experimental results can only represent the samples collected in this study. The data cannot be used to evaluate all RE samples obtained from Jilin province (Huadian, Jilin, Jingyu, Fusong, Linjiang, Tonghua, and Liu He), Heilongjiang province (Shangzhi and Tieli), and Liaoning province (Xinbin). Because *Rana chensinensis* is a wild or semiwild amphibian, the content of active compounds in RE is affected by multiple factors. The quality is not only related to the latitude and longitude of growth but also related to its varieties, growth environment, climate, breeding methods, catching time, drying methods, and other factors. Therefore, it is crucial to control the quality of different batches of RE samples using the quality evaluation method developed in this study.

The ammonia-induced cough test was applied in this study, which is also a feasible method to evaluate the antitussive effect of various TCM. Chuan Bei loquat ointment, a traditional Chinese compound preparation, was selected as the positive control drug. This Chinese patent medicine has a good antitussive effect and is widely used in clinics. It is also a good representative of antitussive drugs. The results suggested that the antitussive effect of RE was similar to that of the Chuan Bei loquat ointment, and both of them had a good antitussive effect.

## 5. Conclusions

In this paper, a simple and feasible HPLC fingerprint quantitative analysis combined with a basic statistical analysis method was established and was successfully applied to the identification of RE origins. The proposed method is a good way to distinguish RE from different origins and to determine the contents of three active compounds simultaneously. In summary, this study provides an effective approach for the quality evaluation of RE and a practical strategy for overall quality control of other animal medicines. At the same time, it was found that RE had a good antitussive effect, which increased the application scope of RE.

## Figures and Tables

**Figure 1:** HPLC reference chromatogram of RE samples.

**Figure 2:** Overlapping chromatograms of RE samples.

**Figure 3:** HPLC chromatograms of mixed standard solution (a) and test solution (b) 2: 1-methyl hydantoin, 14: estradiol, and 29: 4-cholestene-3-one.

**Figure 4:** Dendrogram of hierarchical cluster analysis.

**Figure 5:** The scree plot of HPLC fingerprint.

**Table 1:** The sources and batch numbers of representative RE samples.

Sample no.	Batch no.	Animal species	Collection locations
S1	SZ20180901	*Rana chensinensis*	Shangzhi, Heilongjiang province
S2	TL20180902	*Rana chensinensis*	Tieli, Heilongjiang province
S3	XB20180901	*Rana chensinensis*	Xinbin, Liaoning province
S4	HD20180902	*Rana chensinensis*	Huadian, Jilin province
S5	JL20180901	*Rana chensinensis*	Jilin, Jilin province
S6	FS20180902	*Rana chensinensis*	Fusong, Jilin province
S7	JY20180901	*Rana chensinensis*	Jingyu, Jilin province
S8	LJ20180902	*Rana chensinensis*	Linjiang, Jilin province
S9	TH20181001	*Rana chensinensis*	Tonghua, province
S10	LH20181002	*Rana chensinensis*	Liu He, Jilin province

**Table 2:** The gradient elution conditions of HPLC.

Time (min)	Flow rate (mL/min)	A (%)	B (%)	Column temperature (°C)
0	1.0	0	100	25
6	1.0	0	100	25
10	1.0	25	75	25
24	1.0	80	20	30
30	1.0	86	14	30
30.1	2.0	86	14	30
36	2.0	88	12	30
36.1	0.5	88	12	45
44	0.5	93	7	45
64	0.5	96	4	45
98	0.5	96	4	45
113	1.0	100	0	45

**Table 3:** Relative retention time of common peaks in HPLC chromatograms of RE samples.

Peak no.	S1	S2	S4	S5	S6	S7	S8	S9	S10
1	0.075	0.069	0.069	0.069	0.069	0.070	0.069	0.069	0.069
2	0.115	0.106	0.106	0.107	0.107	0.108	0.107	0.107	0.107
3	0.124	0.119	0.119	0.120	0.120	0.120	0.120	0.120	0.120
4	0.127	0.123	0.124	0.124	0.124	0.124	0.124	0.124	0.124
5	0.130	0.127	0.128	0.128	0.128	0.128	0.128	0.128	0.128
6	0.152	0.149	0.149	0.149	0.149	0.149	0.149	0.149	0.150
7	0.176	0.173	0.173	0.173	0.173	0.173	0.173	0.173	0.174
8	0.191	0.189	0.189	0.189	0.189	0.189	0.189	0.189	0.189
9	0.218	0.218	0.218	0.219	0.218	0.218	0.219	0.219	0.219
10	0.240	0.240	0.240	0.241	0.240	0.241	0.241	0.241	0.241
11	0.248	0.247	0.247	0.247	0.247	0.247	0.247	0.248	0.248
12	0.253	0.253	0.253	0.253	0.253	0.253	0.253	0.254	0.254
13	0.276	0.275	0.275	0.276	0.275	0.276	0.276	0.276	0.276
14	0.300	0.299	0.299	0.299	0.299	0.299	0.299	0.300	0.300
15	0.344	0.343	0.344	0.344	0.343	0.344	0.344	0.344	0.344
16	0.353	0.352	0.352	0.352	0.352	0.352	0.352	0.353	0.353
17	0.381	0.381	0.381	0.381	0.380	0.381	0.381	0.382	0.382
18	0.442	0.440	0.440	0.441	0.440	0.441	0.441	0.442	0.441
19	0.455	0.453	0.453	0.453	0.452	0.453	0.453	0.454	0.454
20	0.515	0.514	0.514	0.514	0.513	0.513	0.513	0.514	0.514
21	0.525	0.523	0.523	0.523	0.522	0.523	0.523	0.524	0.524
22	0.537	0.536	0.536	0.536	0.535	0.535	0.535	0.536	0.536
23	0.556	0.554	0.554	0.554	0.553	0.554	0.554	0.555	0.555
24	0.575	0.574	0.574	0.574	0.573	0.574	0.574	0.574	0.575
25	0.595	0.594	0.594	0.594	0.593	0.594	0.594	0.594	0.595
26	0.609	0.608	0.608	0.608	0.607	0.608	0.608	0.608	0.609
27	0.638	0.636	0.637	0.637	0.636	0.636	0.636	0.637	0.637
28	0.982	0.981	0.982	0.983	0.981	0.982	0.982	0.981	0.982
29 (S)	1.000	1.000	1.000	1.001	1.000	1.000	1.000	1.000	1.000
30	1.056	1.056	1.056	1.056	1.056	1.056	1.055	1.055	1.056
31	1.095	1.094	1.094	1.094	1.093	1.094	1.092	1.093	1.093

**Table 4:** Relative peak areas of common peaks in HPLC chromatograms of RE samples.

Peak no.	S1	S2	S4	S5	S6	S7	S8	S9	S10
1	3.019	3.592	2.567	2.426	2.376	2.118	1.952	2.204	2.452
2	0.752	0.894	0.951	0.857	0.787	1.029	1.098	0.937	1.060
3	0.035	0.120	0.108	0.184	0.054	0.087	0.107	0.102	0.118
4	0.168	0.215	0.241	0.369	0.171	0.273	0.316	0.242	0.269
5	0.681	0.804	0.694	0.787	0.641	0.547	0.614	0.628	0.650
6	0.561	0.886	0.771	0.828	0.605	0.611	0.689	0.707	0.782
7	0.899	1.097	1.050	1.174	0.916	1.156	1.249	0.976	1.082
8	0.498	0.566	0.303	0.445	0.381	0.412	0.386	0.422	0.444
9	7.840	11.150	5.223	8.183	7.056	7.419	7.403	6.689	7.235
10	0.380	0.301	0.260	0.330	0.257	0.369	0.455	0.448	0.365
11	0.359	0.255	0.113	0.181	0.151	0.158	0.164	0.335	0.176
12	0.369	0.293	0.096	0.144	0.204	0.133	0.135	0.073	0.143
13	4.080	4.185	4.685	3.241	2.966	11.142	3.849	6.311	2.957
14	0.197	0.263	0.209	0.170	0.213	0.332	0.286	0.215	0.183
15	2.112	2.462	2.194	2.250	2.021	1.984	1.779	2.142	2.128
16	2.462	2.694	2.197	2.044	1.920	1.917	1.884	2.070	2.089
17	0.999	1.170	0.534	0.501	0.472	0.660	0.564	0.568	0.583
18	11.348	13.949	11.822	12.846	10.559	12.275	12.520	12.366	13.923
19	17.785	18.339	17.817	18.342	16.079	16.708	16.670	18.398	20.057
20	16.871	23.251	19.342	23.308	16.698	19.437	20.018	20.096	22.865
21	8.956	12.732	9.507	11.088	8.357	9.555	9.828	9.423	11.457
22	5.837	7.701	6.125	6.478	5.360	5.456	5.582	5.983	6.678
23	4.543	5.796	4.903	5.491	4.381	4.997	5.085	5.152	5.693
24	0.961	2.449	1.133	1.408	0.957	1.206	1.341	1.101	1.417
25	1.127	1.289	1.161	1.275	1.012	1.209	1.239	1.215	1.386
26	2.104	2.705	2.178	2.478	2.000	2.336	2.385	2.228	2.575
27	0.417	0.525	0.555	0.633	0.363	0.402	0.439	0.422	0.555
28	1.357	1.782	1.555	1.737	1.531	1.547	1.313	1.575	1.709
29 (S)	1.000	1.000	1.000	1.000	1.000	1.000	1.000	1.000	1.000
30	3.601	4.768	3.708	3.979	3.811	4.076	4.028	3.783	4.015
31	1.104	2.463	2.146	3.575	2.055	2.316	1.327	2.370	2.455

**Table 5:** Results of similarity evaluation for 10 batches of RE samples.

Batch no.	S1	S2	S3	S4	S5	S6	S7	S8	S9	S10	Reference
S1	1.000	0.990	0.980	0.969	0.997	0.974	0.993	0.993	0.992	0.994	0.994
S2	0.990	1.000	0.974	0.974	0.993	0.970	0.994	0.987	0.991	0.991	0.992
S3	0.980	0.974	1.000	0.990	0.983	0.967	0.983	0.985	0.985	0.985	0.991
S4	0.969	0.974	0.990	1.000	0.976	0.950	0.977	0.973	0.979	0.977	0.984
S5	0.997	0.993	0.983	0.976	1.000	0.972	0.996	0.994	0.997	0.997	0.997
S6	0.974	0.970	0.967	0.950	0.972	1.000	0.977	0.988	0.967	0.976	0.981
S7	0.993	0.994	0.983	0.977	0.996	0.977	1.000	0.995	0.998	0.998	0.998
S8	0.993	0.987	0.985	0.973	0.994	0.988	0.995	1.000	0.993	0.997	0.997
S9	0.992	0.991	0.985	0.979	0.997	0.967	0.998	0.993	1.000	0.998	0.997
S10	0.994	0.991	0.985	0.977	0.997	0.976	0.998	0.997	0.998	1.000	0.998
Reference	0.994	0.992	0.991	0.984	0.997	0.981	0.998	0.997	0.997	0.998	1.000

**Table 6:** Eigenvalue and variance contribution rate of HPLC fingerprint.

Compound	Eigenvalue	Variance contribution rate (%)	Cumulative variance contribution rate (%)
1	21.063	67.946	67.946
2	2.727	8.797	76.744
3	2.407	7.765	85.509
4	1.746	5.631	90.140
5	1.143	3.686	93.827

**Table 7:** Loading matrices of principal compounds of HPLC fingerprint.

Peak no.	Principal compound (1)	Principal compound (2)	Principal compound (3)	Principal compound (4)	Principal compound (5)
1	0.703	0.691	0.138	0.031	0.016
2 (1-methyl hydantoin)	0.917	−0.194	0.169	0.195	−0.113
3	0.770	−0.116	−0.452	−0.228	0.254
4	0.825	−0.367	−0.235	−0.040	−0.010
5	0.895	0.335	−0.053	−0.126	−0.140
6	0.968	0.160	−0.124	−0.076	0.029
7	0.931	−0.173	−0.011	0.214	−0.127
8	0.781	−0.194	0.269	−0.360	0.142
9	0.580	−0.188	−0.502	0.319	0.199
10	0.523	−0.606	0.450	−0.123	0.062
11	−0.145	−0.101	0.676	−0.571	0.367
12	−0.651	0.633	0.111	0.145	−0.275
13	0.441	−0.345	0.468	0.426	0.286
14 (estradiol)	0.528	−0.356	0.283	0.640	−0.152
15	0.934	0.271	0.143	−0.071	−0.037
16	0.853	0.438	0.270	0.015	0.018
17	−0.012	0.592	0.419	0.369	0.540
18	0.985	−0.053	0.078	0.006	−0.051
19	0.956	0.080	0.191	−0.125	−0.144
20	0.985	−0.065	−0.097	−0.083	0.007
21	0.977	0.061	−0.131	−0.004	0.042
22	0.963	0.235	0.014	−0.068	0.007
23	0.994	−0.042	0.032	−0.034	−0.024
24	0.572	0.160	−0.490	0.276	0.502
25	0.976	−0.083	0.096	−0.027	−0.065
26	0.989	−0.058	−0.006	0.061	−0.040
27	0.916	0.234	−0.177	−0.146	−0.013
28	0.956	0.109	0.012	−0.079	−0.083
29 (4-cholestene-3-one)	0.928	0.058	0.035	0.052	−0.222
30	0.958	0.004	0.067	0.198	−0.089
31	0.772	−0.062	−0.328	−0.285	0.090

**Table 8:** Validation parameters of the three active compounds.

Compound	Standard curve	Linearity range (*μ*g/mL)	*r*	LOQ (*μ*g/mL)	LOD (*μ*g/mL)
1-methyl hydantoin	*Y* = 236.3*X* + 11.36518.768	0.416∼20.80	0.9996	0.56	0.17
Estradiol	*Y* = 61.537*X* − 1.3187	0.385∼19.24	0.9995	0.46	0.11
4-cholesten-3-one	*Y* = 4.7785*X* + 1.2974	1.98∼99.00	0.9997	0.69	0.21

**Table 9:** Results of the recovery test of three active compounds.

Compound	Known content (*μ*g)	Added amount (*μ*g)	Total measured amount (mg)	Recovery rate (%)	Average recovery (%)	RSD (%)
1-methyl hydantoin	10.245	10.06	20.392	100.86	99.44	1.88
	10.486	10.06	20.266	97.21		
	10.412	10.06	20.335	98.64		
	10.437	10.06	20.608	101.11		
	10.412	10.06	20.224	97.54		
	10.462	10.06	20.653	101.31		

Estradiol	7.903	7.96	15.663	97.48	99.13	1.87
	8.089	7.96	16.152	101.29		
	8.032	7.96	15.791	97.48		
	8.051	7.96	15.926	98.93		
	8.032	7.96	15.834	98.02		
	8.070	7.96	16.153	101.54		

4-cholesten-3-one	122.179	121.2	240.714	97.80	98.98	1.77
	125.055	121.2	248.161	101.57		
	124.162	121.2	242.638	97.75		
	124.460	121.2	243.701	98.38		
	124.162	121.2	242.378	97.54		
	124.757	121.2	246.935	100.81		

**Table 10:** Results of quantitative determination (*μ*g/g).

Batch no.	S1	S2	S3	S4	S5	S6	S8	S9	S10
1-methyl hydantoin	5.949	6.231	14.463	8.316	8.703	10.873	11.386	10.524	10.389
Estradiol	6.074	7.154	12.344	6.417	9.168	13.653	5.615	6.106	5.681
4-cholestene-3-one	52.611	80.377	147.602	99.132	77.698	70.147	71.609	104.734	87.441

**Table 11:** Antitussive effect of RE.

Group	Dose	Cough latent period (S)	Cough frequency (S)
Model	—	23.33 ± 5.43	45.44 ± 12.87
Chuan Bei loquat ointment	5.85 ml/kg	39.5 ± 11.39^*∗*^	21.2 ± 5.18^*∗∗*^
A low dose of RE	0.5 g/kg	27.6 ± 11.37	31.5 ± 13.33
A middle dose of RE	1 g/kg	38.6 ± 10.96^*∗∗*^	19.9 ± 6.66^*∗∗*^
A high dose of RE	2 g/kg	40.4 ± 11.21^*∗∗*^	17.4 ± 7.17^*∗∗*^

Results of ammonia-induced cough test are shown ($\bar{X}$ ± *s*, *n* = 10). Compared with the model group, ^*∗*^*P* < 0.05 and ^*∗∗*^*P* < 0.01.

## Data Availability

The main table and figure data used to support the findings of this study are included in the article.
